The article "Mask R-CNN-Oriented Pottery Display and Identification System" was published in 2022. Journal: Comput Intell Neurosci.

# Mask R-CNN-Oriented Pottery Display and Identification System

**DOI:** 10.1155/2022/6288201

**Published:** 2022-06-13

**Authors:** Chuantao Wei

**Affiliations:** Hubei Academy of Fine Arts, Wuhan, Hubei 430205, China

## Abstract

Traditional pottery identification methods are time consuming and costly. In order to cater to more pottery industry needs, we propose a Mask R-CNN-based pottery identification method to build an automatic pottery identification system. We first improve the loss function of Mask R-CNN by using generalized intersection over union loss function, through the pattern of migration learning, to compensate for the disadvantage of a small collective amount of pottery data. For different types of pottery, we use the mask algorithm to enhance the features of the outer contour of the pottery. In addition, we use the minimum external matrix algorithm to accurately extract the outer contour bit pose features of pottery to improve the model's accuracy in recognizing the outer contour of pottery. To meet the testing conditions of pottery, with the support of potters and archaeologists, we make our pottery data set according to pottery categories. The experimental results prove that our method performs best in the comprehensive recognition accuracy of pottery, with the recognition accuracy above 90%. The recognition accuracy is also the best in pottery color decoration and grain decoration, and the grain recognition accuracy stays above 87%, which is better than other pottery recognition methods.

## 1. Introduction

Pottery is an important point in the history of human civilization. As early as the Neolithic era, primitive ancestors had mastered the art of kneading and firing pottery from clay. With the development of human civilization, ancient people continued to research and advance pottery technology, people experimented with the selection of clay types and the mixing ratio with water, and the shape of pottery evolved from practical cooking utensils to works of art. According to archaeologists, for the primitive ancestors, the production and use of pottery were mainly around the development of household items, and in later historical evolution the pottery that was buried in the soil for a long time still maintain the original appearance. The biggest advantage of pottery is that it can be used for a long time and is not easily graded in clay. So much so that pottery was mass produced as a craft in ancient times. After a long history, it has been preserved intact. What has been preserved in pottery is not only the skillful pottery of the generation of craftsmen but also the history and culture of the dynasty. The pottery provides a valuable reference for later archaeologists and antique enthusiasts.

The article "Mask R-CNN-Oriented Pottery Display and Identification System" was published in 2022. Journal: Comput Intell Neurosci.

According to historical records, in the development of ancient pottery, the ancients had an in-depth study of the materials, proportions, fire, and pottery art. The study of pottery in ancient times was a knowledge covering analytical chemistry, literature, art and art, sculpture, handicraft, and so on [1, 2]. Ancient potters had a different understanding of pottery materials, and different dynasties used different mainstream pottery materials, which confirms the different traditional cultures of each dynasty. And the emergence of colored pottery better reflects the lifestyle of ancient people. In addition to the different understanding of carving techniques by the potter of each dynasty, the pottery of each era has a unique shape style. Then later in the emergence of color painting, pottery artists will be celebrity in fusing poetry, songs, and paintings into the pottery, for the pottery to give the soul of culture and art. With the change of dynasties, the development of pottery also showed different characteristics with the rise and fall of dynasties. Pottery reached its artistic pinnacle during the Tang Dynasty, with excellent categories and techniques. Today, archaeologists and pottery enthusiasts have studied ancient pottery to some extent. The different shapes of pottery, different patterns, different carving arts, and so on can determine the culture and lifestyle of the dynasties behind the pottery [3].

From the appearance of the pottery for quality and age judgment is the first stage of pottery identification, a more professional way to identify pottery is to start with the pottery material analysis. In order to obtain more comprehensive information on pottery, archaeologists resort to chemical analysis of pottery materials or physical processing methods. This has significant advantages for the quality analysis of pottery shards, and researchers mostly use multivariate calibration method and metrological analysis in the pottery material analysis data. Such delicate research work is a must for archaeologists, and for the amateur pottery enthusiasts, these pottery identification works are too costly and of low applicability [4, 5]. To make pottery identification more humane and intelligent, some researchers began to try to use machine learning methods for feature learning and classification of pottery categories. Machine learning methods are extremely demanding for manual labeling of features, the labor cost is large, and the recognition accuracy has a great upside. Considering the shortcomings of machine learning methods, some researchers began to try deep learning methods, the fragmented pottery features, and then performed neural network modeling on the fragmented features and achieved the purpose of learning pottery features by updating and iterating the neural network method [6]. The neural network approach can greatly improve the accuracy and speed of pottery recognition. In the subsequent pottery research, to adapt to the feature recognition needs of different pottery, a large number of researchers began to build different neural networks and verify the efficiency of neural networks through a large number of experiments.

The article "Mask R-CNN-Oriented Pottery Display and Identification System" was published in 2022. Journal: Comput Intell Neurosci.

We refer to different neural network models, and finally, we propose a Mask R- –based pottery recognition method to build a pottery automatic recognition system. We improve the loss function of Mask R- by using generalized intersection over union loss function, through the pattern of migration learning, to compensate for the disadvantage of a small collective amount of pottery data. For different types of pottery, we use the mask algorithm to enhance the features of the outer contour of the pottery. To meet the test conditions of pottery, we make our pottery data set according to pottery categories with the support of potters and archaeologists. Finally, we experimentally demonstrate the effectiveness of our method.

The rest of the paper is organized as follows.  Section 2 presents the history and research results of pottery identification research.  Section 3 details the related principles and implementation details of the Mask R- –based pottery recognition network.  Section 4 shows the experimental data sets and the analysis of the experimental results. Finally, Section 5 summarizes our research and reveals some further research work.

## 2. Related Work

The style and texture of pottery are one of the important sources of information about pottery, and the social customs and trade information of the time can be determined based on the appearance and shape of the pottery. In China's Tang Dynasty, potters would carefully select different clays according to the needs of their crafts. Pottery fired from different clays varied greatly in appearance and texture, which is a source of information for archaeologists to identify pottery. The sculptural styles pursued by potters varied from period to period, and the art of hand relief carving took on different styles with the rise and fall of dynasties. In the opinion of decorative researchers, the relief style of pottery represents the artistic trends of the time, which is also a great source of information for pottery identification. By the 1870s, the pottery industry began to take shape, and pottery research was gradually increasing, with pottery analysis and research becoming a popular industry. The traditional pottery identification industry relied heavily on experienced pottery experts, potters, and archaeologists. They use visual perception and empirical judgments to identify types of pottery, techniques, and chronological information. Traditional methods of pottery identification are time consuming and costly. To cater to the needs of more pottery industries, researchers have tried to adopt artificial intelligence to identify pottery information automatically and gradually started to build a pottery feature database to complete the pottery inventory and classification tasks by matching the feature database with additional samples. Considering that pottery artifacts are affected by external environmental factors in the process of preservation, the problem of degradation of pottery relief patterns and its texture occurs. Some researchers try to use deep learning methods to ensure the robustness of the pottery identification system. Some researchers have tried to build a pottery textual feature database by 3D scanning technology and classify the feature database by manual labeling. Some researchers try to seek the relevant factors for pottery classification from different neural network combination strategies, to enhance the sensitivity of neural networks to pottery pattern features.

The article "Mask R-CNN-Oriented Pottery Display and Identification System" was published in 2022. Journal: Comput Intell Neurosci.

To reduce the cost of artifact classification and inventory work, researchers in the literature [7] proposed the idea of building a database of artifact 3D features, and they scanned all the pottery artifacts in inventory in 3D and manually labeled each 3D data. The establishment of the database provided a solid data foundation for the later deep learning model building. In archaeology, for pottery from early times, most of the pottery cannot be preserved intact to this day due to weather and natural environment, and more of the pottery is in the form of shards in our is research. Considering the featured study of pottery shards, literature [8–11] proposed different local feature extraction methods, mainly around the shape and contour of pottery shards, and feature mapping with the data set to obtain pottery sources. Researchers in the literature [12–17] also established a separate pottery color database and material features database to compensate for the lack of color features and material features in the previous data set. In the literature [18–20], to distinguish the details of pottery decorations, researchers established a database of pottery pattern reliefs, which mainly focuses on different pottery decorations for information annotation.

Researchers in the literature [21] found in the study of pottery shards that the appearance profile of the shard can influence the expert's overall judgment of the surface model of the pottery. The curvature of the appearance of the sherd profile, axis detection parameters, symmetry, and bending strength are all factors that must be considered in sherd studies in pottery sherd matching work [22]. In the literature [18], an analogical approach was proposed in the study of pottery decoration, where the researcher correlated the classification of pottery with the color decoration and relief patterns of pottery to build a 2D pottery decoration corpus and mapped the pottery shard decoration features to the database as a way to match to the information of the original pottery. Since the 2D corpus is not effective in 3D relief decoration, researchers in the literature [19] tried to integrate computer vision techniques into the identification of pottery reliefs, which have multiple parallel patterns or irregular patterns in numerous archaeological finds, and each pattern requires an independent database to be associated with it. Therefore, researchers in the literature [20] proposed a convolutional neural network-based pottery decorative template matching method, where they first preprocessed the pottery shards, then laser scanned the shards to obtain a model of the shard carving patterns, then segmented the model with hyperbolic pattern features, and finally trained independent segmentation features with convolutional neural networks to obtain a pottery decorative template identification model.

The article "Mask R-CNN-Oriented Pottery Display and Identification System" was published in 2022. Journal: Comput Intell Neurosci.

There are many different types of pottery, from domestic pottery items to pottery craft artworks, each with a unique pattern of decoration. The design of specialized pottery identification models for different categories of pottery is the mainstream research philosophy of researchers today. To ensure a faster pottery classification at a later stage, each pottery is manually labeled at the pottery laser scanning stage, and the source of the labeled information behind the pottery is directly accessible when extracting the pottery 3D model. Researchers in the literature [23] were inspired by the pyramid histogram and used SVM models to classify the visual features of pottery scans. Since there is a lot of room for optimization of machine learning methods in terms of accuracy and speed. Researchers in the literature [24] proposed an AlexNet-based pottery identification model. Researchers in the literature [25] built a pottery identification unit in the VGG11 network inspired by Google neural network to achieve pottery feature identification. The researchers in [26] proposed a pottery identification method based on ResNet18 and verified the effectiveness of the method through experiments.

The article "Mask R-CNN-Oriented Pottery Display and Identification System" was published in 2022. Journal: Comput Intell Neurosci.

## 3. Method

### 3.1. Basic Network

We investigated many neural network algorithms and performed experimental validation, and finally, we chose Mask R-CNN as the network base. Mask R-CNN belongs to the instance segmentation algorithm, and in pottery category identification, Mask R-CNN can perform pottery feature acquisition from pixel level and also instance segmentation from the pottery 3D model and take different colors to mask over the target features [27]. Mask R-CNN belongs to a two-stage algorithm, where the first stage scans the sample data to generate weight extraction candidate regions and the second stage outputs target class masks on a recurrent convolutional neural network branch. In the 3D space, the information contained in each target mask is extracted in a refined way for the whole tau, which can cover the recognition target accurately [28].

Mask R-CNN is obtained by optimizing based on R-CNN, which is a network to mine more feature information from the target, and the authors use a region generation network to build a feature pyramid. To prevent overfitting by stacking the network too much, Mask R-CNN borrowed the VGG network proposed by Google, and the authors proposed the ResNet network based on the VGG network with the adaptive improvement of Mask R-CNN, which has the biggest advantage of using ROIAlign instead of the region of interest pooling. The structure of the Mask R-CNN network is shown in Figure 1.

### 3.2. Region Proposal Network

The region proposal network (RPN) is the core of the Mask R-CNN network. Its network structure is shown in Figure 2. At the pixel level, RPN will traverse each pixel point, and each pixel point will generate *K* anchor frames of different sizes accordingly, and each anchor frame will correspond to a background label independently. When the intersection ratio between the target real frame and the predicted frame is greater than the predefined maximum threshold, the predicted frame will be considered as the foreground. When the intersection ratio is less than the predefined minimum threshold, it will be considered as the background. When the intersection ratio is between the maximum and minimum thresholds, the prediction frame is considered the no-target case. The final output of RPN has 4K dimensions of location information and 2*K* dimensions of final output feature information. R-CN

Each target prediction box generated by the RPN network will exist in the pattern of Figure 3, where the red box represents the initial prediction box, the green box represents the real box, and the blue box represents the final prediction box.

If the pixel position of each anchor box needs to be determined, it needs to be calculated using the border regression algorithm, and the area between the prediction box and the real box obtained by the algorithm is the prediction generation area of the target. Each box has corresponding parameter coordinates [*x*, *y*, *w*, *h*], where *x* and *y* denote the pixel coordinates of the top left corner of the anchor box, *w* denotes the width of the anchor box, and *h* denotes the height of the anchor box. After the initial prediction box is feature mapped, the final prediction box then has the following mathematical expression.

(1) $$\begin{array}{c} f\left(P_{x},P_{y},P_{w},P_{h}\right)=\left({\overset{⌢}{G}}_{x},{\overset{⌢}{G}}_{y},{\overset{⌢}{G}}_{w},{\overset{⌢}{G}}_{h}\right)\approx \left(G_{x},G_{y},G_{w},G_{h}\right). \end{array}$$

In the feature extraction process of the RPN network, the prediction frame will be automatically scaled according to the size of the real frame, and then the translation convolution will be calculated.

(2) $$\begin{array}{c} {\hat{G}}_{x}=P_{w}d_{x}\left(P\right)+P_{x},\\ {\hat{G}}_{y}=P_{h}d_{y}\left(P\right)+P_{y},\\ {\hat{G}}_{w}=P_{w}\exp\left(d_{w}\left(P\right)\right),\\ {\hat{G}}_{h}=P_{h}\exp\left(d_{h}\left(P\right)\right), \end{array}$$

where *d*_*∗*_(*P*) denotes the initial predicted value and the true value is known, assuming *d*_*∗*_(*P*)=*w*_*∗*_^*T*^Φ_5_(*P*), Φ_5_(*P*) denotes the feature vector of the input initial value, and *w* represents the parameter to be learned, and we also use the least-squares method to reduce the gap between the predicted value and the true value.

(3) $$\begin{array}{c} \text{Loss}=\sum_{i}^{N}{\left(t_{*}^{i}-{\hat{w}}_{*}^{T}f_{5}\left(P^{i}\right)\right)}^{2}. \end{array}$$

*W* is obtained by bringing LOSS to a minimum value. The expression *k* of the ROI region can be obtained through the RPN network.

(4) $$\begin{array}{c} W={\text{argmin}}_{w_{*}}\overset{N}{\underset{i}{\sum }}{\left(t_{*}^{i}-{\hat{w}}_{*}^{T}\phi_{5}\left(P^{i}\right)\right)}^{2}+\lambda {\hat{w}}_{*}^{2},\\ k=k_{0}+\log_{2}\left(\frac{\sqrt{wh}}{224}\right), \end{array}$$

where 224 denotes the pixel size of the target and *k*0 denotes the layer where the ROI with area *w* × *h* = 224 × 224 is located. In addition, the value of *k* needs to be kept as an integer so that the large-scale ROI can extract large target features smoothly even on the low-resolution feature map, and the small-scale ROI can extract small target features from the high-resolution feature map.

The article "Mask R-CNN-Oriented Pottery Display and Identification System" was published in 2022. Journal: Comput Intell Neurosci.

### 3.3. Loss Function Optimization

The loss function of the Mask R-CNN network contains the classification loss function and regression loss function. The loss function of the Mask R-CNN model has an additional mask branch compared to the R-CNN network, and the mathematical expression is as follows:

(5) $$\begin{array}{c} L=L_{cls}+L_{\text{box}}+L_{\text{mask}}, \end{array}$$

where *L*_*cls*_ denotes the classification loss function, *L*_box_ denotes the regression loss function, and *L*_mask_ denotes the mask loss function. Each independent loss function uses the *L*1 function and *L*2 function in predicting the edges and the true edges. Most of the loss functions take the cross-merge ratio as a constraint for calculating the overlap value between the prediction frame and the real frame, but the cross-merge ratio cannot reflect the form of overlap between the prediction frame and the real frame, resulting in the distance between the two cannot be accurately estimated, so we propose the GIOU method, which is calculated as shown below.

(6) $$\begin{array}{c} IOU=\left|\frac{A\cap B}{A\cup B}\right|,\\ GIOU=IOU\;-\;\frac{\left|C/\left(A\cup B\right)\right|}{\left|C\right|}. \end{array}$$

Assume two arbitrary polygons *A* and *B*. *C* denotes the smallest closed object from the overlapping part of *A* and *B*. Generalized intersection over union (GIOU) is similar to the calculation of IOU with scale invariance. The value of IOU is always greater than the value of GIOU. When the prediction frame is far away from the real frame, the merge between them increases and GIOU decreases. The problem of not being able to judge the relative position between the predicted frame and the real frame can be solved by the way of this and the other.

### 3.4. Transfer Learning

Different deep neural networks have different training settings and different data set training durations. Our research focuses on the type identification of pottery, and pottery database construction is a huge project. The collective amount of pottery data that has been constructed at present is not large and the number of samples is limited. To verify the effectiveness of our method in a limited sample, we proposed a transfer learning method. We also refer to the migration model of feature parameters mentioned in the literature [29], which reduces the model training time and saves the cost of computer computing power. Migration learning contains the source domain and target domain in the mathematical expression, and their mathematical definitions are as follows:

(7) $$\begin{array}{c} D\left(S\right)=\left\{x,P\left(x\right)\right\},D\left(t\right)=\left\{x,P\left(x\right)\right\}, \end{array}$$

where *D*(*S*) denotes the Source domain, *D*(*t*) denotes the Target domain, *x* denotes the feature interval of the domain, and *P*(*x*) represents the edge probability distribution corresponding to the feature space. We adopt the pottery data set as the auxiliary sample *X*_*a*_ and the pottery enhancement data set as the spatial sample *X*_*b*_ and assume that *Y* = {0, 1, 2, 3}, which contains 4 types of pottery as samples, the training data *T* and the test data S satisfy the following equations.

(8) $$\begin{array}{c} T\subseteq \left\{\left(X=X_{b}UX_{a}\right)Y\right\},\\ S=\left\{\left(x_{i}^{t}\right)\right\},\\ T_{a}=\left\{\left(x_{i}^{a},c\left(x_{i}^{a}\right)\right)\right\},\\ T_{b}=\left\{\left(x_{j}^{b},c\left(x_{j}^{b}\right)\right)\right\}, \end{array}$$

where the training set *T* is divided into two subsets *T*_a_ and *T*_b_. *x*_*i*_^*t*^ ∈ **X**_*b*_, where *i* = 1, 2,…, *k*, *x*_*i*_^*a*^ ∈ **X**_*a*_, where *i* = 1, 2,…, *n,x*_*j*_^*b*^ ∈ **X**_*b*_, where *j* = 1, 2,…, *m.* In the migration learning design of the pottery recognition network, we first normalize the pottery data set so that the data set satisfies a linear distribution. Then we update the sample weights of the pottery data set by using the public data set as network pretraining and comparing the pottery training results for error rate reset. For the correctly trained samples, we reduce the correlation weights, and for the incorrectly trained samples, we take the means of weight superposition. All pottery samples are updated iteratively until the error rate reaches within the specified range. In the pretraining process, we use ResNet as the base network to train the pottery for a phase of parameter calibration, adjust the parameters, and set the weights for the Mask R-CNN network according to the training results [30]. The detailed process of transfer learning is shown in Figure 4.

The article "Mask R-CNN-Oriented Pottery Display and Identification System" was published in 2022. Journal: Comput Intell Neurosci.

### 3.5. Pottery Identification System

Referring to a large number of pottery recognition studies, we choose to base on the Mask R-CNN network. Based on this, we introduced the GIOU loss function to enhance the extraction ability of the model on the generalized features of the target, and we chose Compute Unified Device Architecture to accelerate the model computation ability. To improve the pottery identification system, we added a laser scanner as the data source center of computer vision. The pottery scanning data samples are convolved to get the pyramid feature layer, and then the candidate regions are extracted on the feature layer, and the candidate regions are pooled and convolved to extract features. We introduce the GIOU loss function after the pooling layer and set 3 threshold criteria for the GIOU loss function and finally get the type features, grain location, and shape features of pottery by iterative training of pottery feature update and CUDA model acceleration. The model gets the pottery plane position after recognizing the pottery, but the laser scanner input is the three-dimensional information of the pottery, the pottery carving information requires spatial position features and angle features, and the bit pose estimation method mainly collects the pottery texture, edge shape, and other features. In the real environment, the imaging quality will be degraded due to factors such as lighting and texture, and the above geometric feature-based method is susceptible to great influence.

The article "Mask R-CNN-Oriented Pottery Display and Identification System" was published in 2022. Journal: Comput Intell Neurosci.

After the traditional deep learning target detection algorithm recognizes the pottery, it will be seriously affected by the lighting, texture, and complex background, etc., which leads to the difficulty of edge extraction and has a big impact on the pottery 3D feature prediction because there is no reinforcement of the edge information. Our method can also perform pixel-level feature segmentation for pottery in a complex environment using the mask algorithm. The mask reinforces the pottery edge features and can better perform the task of locating the pottery 3D boundaries, and the edges of the already segmented image are extracted using the mask to generate pixel-level masks. We extract the mask obtained from the algorithm separately to generate the mask map and use the minimum external moment algorithm to accurately extract the pottery angle information, which can be used with the coordinate information obtained from the target recognition to obtain the pottery carving texture features [31]. The details of the pottery recognition system are shown in Figure 5.

## 4. Experiment

### 4.1. Data Set

There is no systematic pottery data set in the current pottery identification research.

To validate our pottery identification method, we made our pottery data set with the support of potters and archaeologists. To standardize the types of pottery, we set five major pottery categories at the early stage of pottery data set production, namely color pottery, faience, painted pottery, stamped pottery, and glazed pottery. Color pottery is mainly made of clay, ming, and material mixed with water in appropriate proportions, then shaped, dried, and fired. Faience is pottery made with iron oxide and manganese oxide as coloring elements. Painted pottery is pottery made by painting colors on the finished product after firing. Stamped pottery is pottery made by laying the clay on a bamboo mat or linen cloth and printing a pattern or cloth pattern. Glazed pottery is a compound of lead as an accelerant, after several firings of pottery, pottery external glaze is not only colorful but also not easy to fall off, commonly used in the language of crafts pottery production. According to the five major categories of pottery, we made different pottery data sets, respectively. The detailed data set information is shown in Table 1.

The article "Mask R-CNN-Oriented Pottery Display and Identification System" was published in 2022. Journal: Comput Intell Neurosci.

### 4.2. Experimental Settings

To ensure the independence and stability of the pottery identification system, we configured an independent host computer for the system, and all the integrated systems were developed with the host computer as the platform. In our experiments, we mainly configured the experimental environment with the Anaconda system. Considering the different requirements of the vision system and the pottery identification system for the programming environment, we configured multiple programming environments on the host computer to suit different needs. In the construction of the pottery identification neural network, we mainly use TensorFlow as the main framework. With the support of TensorFlow's powerful community module, our pottery identification network can be successfully built. The detailed training parameters are shown in Table 2.

For the method testing efficiency metrics, we chose recall (*R*) and precision (*P*) as general evaluation metrics. Where *X*_TP_ denotes correctly identified pottery, *X*_FN_ denotes unidentified pottery, and *X*_FP_ denotes misclassified pottery. The detailed mathematical calculation is shown below.

(9) $$\begin{array}{c} R=\frac{X_{TP}}{X_{TP}+X_{FN}},\\ P=\frac{X_{TP}}{X_{TP}+X_{FP}}. \end{array}$$

### 4.3. Analysis of Experimental Results

To verify the effectiveness of our pottery recognition system, we compared machine learning methods and deep learning methods. Among the machine learning methods, we chose the SVM [32] algorithm, and among the deep learning algorithms, we chose the SSD algorithm [33] and the Faster R-CNN [34] algorithm. To ensure the independent validation relationship among the methods, we conducted five sets of experiments during the training process to independently validate the recognition efficiency of each group of methods for different classes of pottery. The detection results of each method are directly input into the statistical calculation part of the data set, and the final evaluation results are obtained by balancing the total number and quality of the data set. In the first phase of experiments, we validated all pottery data sets and compared the efficiency of our method with other methods, and the experimental results are shown in Table 3.

The *X*_TP_ in the experiment denotes the recognition efficiency per 500 pottery samples. From the experimental results in Table 3, it can be seen that the SVM method has the highest number of pottery misidentifications, accounting for one-fifth of the total. The recall rate is only 63.5% and the accuracy is not high. The pottery recognition efficiency is slightly better compared to SSD and Faster R-CNN methods, but there is still room for optimization. Our method has only 7 false identifications, and the pottery recognition accuracy reaches 98.3%. It is superior to other methods, which shows the superiority of our method in the first phase of experimental validation. In the second phase of the experiment, we verified the recognition accuracy of each class of pottery separately. Before the experiment started, we performed preprocessing operations on the data of no class of pottery to standardize the input format and sample frame rate of pottery to prevent the influence of data differences on the experimental results. The results of the second stage experiments are shown in Table 4.

The article "Mask R-CNN-Oriented Pottery Display and Identification System" was published in 2022. Journal: Comput Intell Neurosci.

From the experimental results of the second stage, it is clear that the recognition accuracy of traditional machine learning methods in various types of pottery is between 65% and 76%, which does not meet the practical needs in pottery classification work. Both SSD and Faster R-CNN methods keep the pottery recognition accuracy between 80% and 90%, and the pottery recognition efficiency is more stable. Our methods both maintain above 90% in pottery recognition accuracy, which proves the superiority of our methods in the second phase of experimental validation.

In the third phase of the experiment, to verify the recognition accuracy of the pottery identification system for three-dimensional pattern decoration and color decoration, we divided the pottery into two categories: pattern-decorated pottery and color-decorated pottery, where pattern-decorated pottery contains stamped and glazed pottery, and the remaining three categories are regarded as color-decorated pottery. The experimental results are shown in Table 5.

From the experimental results of the third stage, it is clear that all the methods have higher recognition accuracy in color pottery decoration than in pattern pottery decoration. Because patterned pottery decoration requires high 3D features, the traditional SVM method cannot capture pottery 3D features. SSD and Faster R-CNN outperform the SVM method in capturing 3D features, but still need to be optimized. Our method is the best performer in both color pottery decoration recognition and pattern pottery decoration recognition, and the pottery recognition accuracy is better than SSD and Faster R-CNN. It proves the effectiveness of our method in the third stage of experimental validation.

## 5. Conclusion

In this paper, we propose a Mask R-CNN-based pottery recognition method and build a pottery automatic recognition system. We first improve the loss function of Mask R-CNN by using generalized intersection over union loss function, through the pattern of migration learning, to compensate for the disadvantage of a small collective amount of pottery data. For different types of pottery, we use the mask algorithm to enhance the features of the outer contour of the pottery. In addition, we use the minimum external matrix algorithm to accurately extract the outer contour bit pose features of pottery to improve the model's accuracy in recognizing the outer contour of pottery. To meet the testing conditions of pottery, with the support of potters and archaeologists, we make our pottery data set according to pottery categories. The experimental results prove that our method performs best in the comprehensive recognition accuracy of pottery, with the recognition accuracy above 90%. The recognition accuracy is also the best in pottery color decoration and grain decoration, and the grain recognition accuracy is maintained above 87%. It proves that our method performs well in both feature capture at the two-dimensional level and three-dimensional level of pottery. Compared with traditional machine learning methods and deep learning methods, our method has higher recognition accuracy and better stability.

The article "Mask R-CNN-Oriented Pottery Display and Identification System" was published in 2022. Journal: Comput Intell Neurosci.

Compared with machine learning methods and deep learning methods, our method still has much room for improvement in recognition accuracy and recognition efficiency. Although it performs the best in the experiment of grain decorated pottery recognition. In future research, we will try to add a generative adversarial neural network as an auxiliary classification in the adversarial network to optimize the recognition of spatial pattern features during pottery pattern feature segmentation and improve the robustness and generalization of the network.

## Figures and Tables

**Figure 1:** Mask R-CNN network.

**Figure 2:** The principal structure of the region proposal network.

**Figure 3:** Region generation principle.

**Figure 4:** Transfer learning process.

**Figure 5:** Pottery recognition system.

**Table 1:** Pottery data set classification and quantity.

	Train	Test	Total
Color pottery	15531	2011	17542
Faience	17323	1964	19287
Painted pottery	18036	2311	20347
Stamped pottery	16634	3002	19636
Glazed pottery	15321	1906	17227

**Table 2:** Parameter settings.

Parameter	Value
Learning rate	0.01
Decay rate	0.0001
Momentum	0.9
Epoch	70
Iterations	1000
Dropout rate	0.5

**Table 3:** Comparison of pottery identification experiments by different methods.

Method	*X*_TP_	*X*_FP_	*X*_FN_	*R* (%)	*P* (%)
SVM	293	102	85	63.5	76.8
SSD	365	67	53	87.3	84.4
Faster R-CNN	383	35	29	90.9	91.6
Ours	463	7	5	97.1	98.3

The article "Mask R-CNN-Oriented Pottery Display and Identification System" was published in 2022. Journal: Comput Intell Neurosci.

**Table 4:** Comparison of recognition accuracy of different categories of pottery.

Method	Color pottery (%)	Faience (%)	Painted pottery (%)	Stamped pottery (%)	Glazed pottery (%)
SVM	70	73	76	69	65
SSD	82	85	86	80	79
Faster R-CNN	85	90	92	83	83
Ours	95	97	98	90	91

**Table 5:** Comparison of recognition accuracy of pottery decoration by different methods.

	Pattern decoration pottery (%)	Color decoration pottery (%)
SVM	65	72
SSD	72	78
Faster R-CNN	75	83
Ours	87	94

## Data Availability

The data set can be accessed upon request.
